# Autocrine motility factor receptor promotes the proliferation of human acute monocytic leukemia THP-1 cells

**DOI:** 10.3892/ijmm.2015.2267

**Published:** 2015-06-30

**Authors:** YINGCHAO WANG, LINA MA, CHUNMEI WANG, GUANGYAO SHENG, LEI FENG, CHUYUN YIN

**Affiliations:** Department of Pediatrics, the First Affiliated Hospital of Zhengzhou University, Zhengzhou, Henan 450000, P.R. China

**Keywords:** autocrine motility factor receptor, Rho-associated, coiled-coil containing protein kinase 2, acute monocytic leukemia, THP-1, cyclin D1

## Abstract

The aberrant activation of autocrine motility factor receptor (AMFR) has been implicated in several types of human cancer. The present study aimed to elucidate the effect of AMFR on the regulation of proliferation in an acute monocytic leukemia cell line, THP-1. THP-1 cells were transfected with AMFR-targeted small interfering (si)RNA and a plasmid encoding a truncated AMFR, AMFR-C, (pcDNA3.1-AMFR-C). The mRNA and protein levels of AMFR and the downstream targets, rho-associated, coiled-coil containing protein kinase 2 (ROCK2), cyclin D1, and B-cell lymphoma (Bcl)-2, were measured using reverse transcription-quantitatibe polymerase chain reaction and immunoblot analyses. The effects on cell cycle and apoptosis were investigated using flow cytometry. The present study successfully established the knockdown of AMFR and expression of AMFR-C in the THP-1 cells. Downregulation of AMFR induced cell cycle arrest at the G_0_/G_1_ phase, and increased apoptosis of the THP-1 cells (all P<0.05). The AMFR siRNA increased the percentage of early apoptotic cells between 3.88±1.43 and 19.58±4.29% (P<0.05). The expression levels of ROCK2, cyclin D1 and Bcl-2 were reduced by the downregulation of AMFR and enhanced by overexpression of AMFR-C. In conclusion, AMFR appears to be crucial for the proliferation of the THP-1 acute monocytic leukemia cell line. Therefore, AMFR may represent a potential target for the treatment of acute monocytic leukemia.

## Introduction

Acute monocytic leukemia is a form of acute myelogenous leukemia (AML), which is a group of malignant disorders characterized by the abnormal accumulation of immature cells of the myelomonocytic lineage in the bone marrow and periphery (1). Although chemotherapy can induce complete remission in 80–90% of children diagnosed with acute monocytic leukemia (2,3), relapse occurs in 30–40% of patients (4), thus further characterization of the pathogenesis of monocytic leukemia may facilitate the development of novel therapies.

The activation of autocrine motility factor receptor (AMFR) by autocrine motility factor (AMF), a motility-stimulating protein that is secreted by tumor cells, has been demonstrated to be important in proliferation, apoptosis and tumor migration (5–12). The stimulation of AMFR by AMF can trigger a signaling cascade, dependent on protein kinase C, and promotes the activation and upregulation of Rho-like GTPase, RhoA and RhoC (13,14). Rho-associated, coiled-coil containing protein kinase 2 (ROCK2), a member of the RhoC family, also serves as a molecular switch in several cellular functions, including proliferation, apoptosis and metastasis (14,15).

The overexpression of AMFR has been observed in several types of human cancer, including esophageal carcinoma, hepatocellular carcinoma, breast carcinoma, pulmonary cancer and melanoma (16–23), and the expression of AMFR has been found to be significantly correlated with more advanced tumor stage and decreased survival rates in liver, breast, lung and esophageal cancer (16–23). The overexpression of ROCK2 has also been reported in several types of solid tumor (24–26). The majority of previous studies investigating AMFR and ROCK2 have focused on solid tumors, and only one demonstrated that the expression of AMFR was associated with progression in chronic lymphocytic leukemia (27).

In the present study, the effects of knockdown and overex-pression of AMFR in the THP-1 human monocytic cell line, derived from an acute monocytic leukemia patient (27) were investigated. AMFR appeared to be crucial for the proliferation of the THP-1 acute monocytic leukemia cell line. It was observed that the downregulation of AMFR induced cell cycle arrest and increased the apoptosis of the THP-1 cells, In addition, the expression levels of ROCK2, cyclin D1 and B-cell lymphoma (Bcl)-2 were reduced by downregulation of AMFR and enhanced by overexpression of AMFR-C.

## Materials and methods

### Cell culture

The human acute monocytic leukemia cell line, THP-1, was purchased from the Shanghai Institute of Cell Resource Center of Life Science (Shanghai, China), and cultured in RPMI-1640 medium supplemented with 10% fetal bovine serum (FBS) (GE Healthcare Life Sciences, Logan, UT, USA) and 100 U/ml penicillin-streptomycin (Life Technologies, Grand Island, NY, USA), as growth medium, in a humidified incubator at 37°C with 5% CO_2_.

### Overexpression and knockdown of AMFR in THP-1 cells

The pcDNA3.1-AMFR-C plasmid, encoding a 50kDa truncated form of AMFR (AMFR-C), was provided by Professor Le-xun Xue (16), and transfected into the THP-1 cells by electroporation using an Electro Cell Manipulator (BTX Harvard Apparatus, Holliston, MA, USA). Briefly, 1×10^7^ THP-1 cells were cultured in penicillin-streptomycin-free RPMI-1640 medium at 37°C for 24 h prior to transfection. The cells were harvested, washed twice with phosphate-buffered saline (PBS) and resuspended in 0.8 ml medium containing 20% FBS. The cell suspension was divided into two electro cell cups, to which 15 *µ*g of the pcDNA3.1 or pcDNA3.1-AMFR-C plasmids were added. Following mixing for 5 min, a current of 200 V and 950 UF was applied at 37°C for 5–10 min, and the cell suspension was transfered into a 100 ml culture flask containing 10 ml growth medium. The cells were harvested 72 h after transfection.

Subsequently, the THP-1 cells were transiently transfected with AMFR siRNA (cat. no. sc-43809; Santa Cruz Biotechnology, Inc.) or scrambled siRNA (cat. no. sc-36869; Santa Cruz Biotechnology, Inc.), a non-target fluorescein isothiocyanate (FITC)-conjugated control, in small interfering (si)RNA transfection reagent (car. no. sc-29528; Santa Cruz Biotechnology, Inc., Santa Cruz, CA, USA), according to the manufacturer's instructions, as previously described (28,29). Transfection was detected using fluorescent microscopy (ECLIPSE TE2000-U; Nikon Corporation, Tokyo, Japan), and a transfection efficiency of 60–70% was achieved.

### Reverse transcription-quantitative polymerase chain reaction (RT-qPCR)

At 24, 48, 72 and 96 h post-transfection, total RNA was extracted from the THP-1 cells using an RNA Prep Pure Cell kit (Tiangen Biotech Co., Ltd., Beijing, China). The RNA purity was determined according to the absorbance at 260 and 280 nm (A260/280; ultraviolet spectrophotometry, U-2001; Sartorius Corporation, Göttingen, Germany) and the RNA was reverse transcribed into cDNA using a RevertAid™ First Strand cDNA Synthesis kit (MBI Fermentas, Inc., Burlington, ON, Canada), according to the manufacturer's instructions. The expression of AMFR was detected by qPCR using a SYBR-Green kit (Tiangen Biotech Co., Ltd.) with the following primers (Sangon Biotech, Shanghai, China): Forward 5′-GTCAGGGAAGAACATCAAGGAG-3′ and reverse 5′-GGGGAAACATCTCTTGAATCTG-3′. β-actin, used as an internal control, which was detected uising the following primers: Forward 5′-CCCATCTATGAGGGTTACGC-3′ and reverse 5′-TTTAATGTCACGCACGATTT-3′. The qPCR was performed on a 7300 Real-Time PCR System (Applied Biosystems, Foster City, CA, USA) under the following thermal cycling conditions: Initial heating at 95°C for 5 min, followed by 35 cycles of 94°C for 30 sec, 60°C for 30 sec and 72°C for 30 sec, with a final dissociation stage at 95°C for 15 sec, 60°C for 30 sec and 95°C for 15 sec. The threshold cycle (Ct) value was defined as the number of PCR cycles in which the fluorescence signal exceeded the detection threshold value. The relative gene expression was analyzed using the 2^−ΔΔCt^ method.

### AMFR, AMFR-C, ROCK2, cyclin D1 and Bcl-2 immunoblotting

At 72 h post-transfection, the THP-1 cells were lysed in cold lysis buffer (Beyotime Institute of Biotechnology, Beijing, China), centrifuged at 13,400 × g for 5 min at 4°C and the supernatant was collected. The protein concentration in this supernatant was determined using the Bradford method [bovine serum albumin (BSA) was used at 9 different concentrations (0.25, 0.5, 1, 1.5, 2, 3, 4, 5 and 6 mg/ml) to prepare a protein standard. After diluting the protein standards, the stock dye reagent was prepared (500 mg Coomassie Blue was dissolved in 500 ml methanol and was added to 100 ml phosphoric acid and 50 ml ddH_2_O) that was diluted in 8 ml ddH_2_O. Two milliliters of dye reagent were added to each tube of protein standard and incubated at room temperature for at least 5 min. The absorbance of the protein standards and experimental samples was carried out by spectrophotometry (Bausch and Lomb, Berlin, Germany) at 595 nm and, finally, a standard curve was plotted]; and the protein was separated using 10% SDS-PAGE (ST628; Beyotime Institute of Biotechnology), and then transferred onto a polyvinylidene difluoride membrane (Beyotime Institute of Biotechnology) using semi-dry transfer (POWER/RAC200; Bio-Rad Laboratories, Inc., Hercules, CA, USA). The membranes were blocked at 4°C overnight in 5% skimmed milk in Tris-buffered saline containing 0.05% Tween-20 (TBST; ST825; Beyotime Institute of Biotechnology), and then incubated with rabbit anti-human AMFR polyclonal antibody (sc-33541) to identify the AMFR and AMFR-C proteins, rabbit anti-human ROCK2 polyclonal antibody (sc-5561), mouse anti-human cyclin D1 monoclonal antibody (sc-70899), mouse anti-human Bcl-2 monoclonal antibody (sc-7382) or goat anti-human β-actin polyclonal antibody (sc-1616) (all Santa Cruz Biotechnology, Inc.) at room temperature for 2 h. The membranes were then washed three times with TBST, and incubated with the appropriate horseradish-peroxidase-conjugated secondary antibody (Zhongshan Golden Bridge Biotechnology Co., Ltd., Beijing, China). The primary antibodies were diluted at 1:200. The secondary antibodies were diluted at 1:1,000. The membranes were developed using Western Blotting Luminol Reagent (sc-2048; Santa Cruz Biotechnology, Inc.), according to the manufacturer's instructions. Images were captured using Image Scanner III (Amersham Biosciences, Uppsala, Sweden).

### Flow cytometric analysis of cell cycle distribution

The THP-1 cells were harvested 72 h after transfection and washed twice with PBS. The supernatant was discarded and replaced with 1 ml 70% cold methanol. Following incubation at 4°C for at least 12 h, the cells were washed with PBS and stained with 5% propidium iodide (PI; Beyotime Institute of Biotechnology), supplemented with RNase, and incubated in the dark at room temperature for 30 min. The DNA content was analyzed using flow cytometry (FACSCalibur; BD Biosciences, San Jose, CA, USA), with 10,000 events recorded for each sample. The percentage of cells in the G0/G1, S and G2/M phases were determined using CellQuest software (version 3.3; BD Biosciences).

### Flow cytometric analysis of apoptosis using annexin V-FITC/PI staining

At 72 h post-transfection, apoptosis was detected using an Annexin V-FITC Apoptosis Detection kit (Beyotime Institute of Biotechnology), according to the manufacturer's instructions. Briefly, the THP-1 cells were harvested, washed twice with cold PBS and resuspended in binding buffer (included in the Annexin V-FITC Apoptosis Detection kit) at 5×10^5^ cells/ml. Annexin V-FITC (5 *µ*l) was added to 195 *µ*l of the cell suspension, which was mixed and incubated for 10 min in the dark at room temperature. The cells were washed with binding buffer and centrifuged at 250 × g at room temperature. The supernatant was discarded and the cell pellet was resuspended in 190 *µ*l binding buffer. PI (10 *µ*l) was added, and the cells were vortexed and analyzed using flow cytometry (FACSCalibur; BD Biosciences), with 10,000 events recorded for each sample. Early apoptotic events were identified as annexin V-positive, PI-negative staining, determined using CellQuest software (BD Biosciences).

### Statistical analysis

Data were analyzed using the SPSS 18.0 software package (SPSS, Inc., Chicago, IL, USA). Data are presented as the mean ± standard deviation from three independent experiments. Differences between groups were analyzed using an independent samples t-test or one-way analysis of variance, with a least significant difference test for post-hoc analysis. P<0.05 was considered to indicate a statistically significant difference.

## Results

### Expression of AMFR, AMFR-C and ROCK2 in THP-1 cells transfected with pcDNA3.1-AMFR-C

The expression of AMFR and ROCK2 were detected in the THP-1 cells (Fig. 1A). At 72 h post-transfection with the pcDNA3.1-AMFR-C plasmid, AMFR expression was detected in the THP-1 cells transfected with pcDNA3.1-AMFR-C, but not in those transfected with the pcDNA3.1 control plasmid (Fig. 1B).

### siRNA knockdown of the expression of AMFR in THP-1 cells

The mRNA expression of AMFR was significantly decreased in the THP-1 cells transfected with AMFR siRNA for 24, 48, 72 and 96 h, compared with those transfected with scrambled siRNA (P<0.05), and the lowest expression level of mRNA was measured at 72 h post-transfection with AMFR siRNA (Fig. 2A). The protein level of AMFR was also significantly decreased 72 h after AMFR siRNA transfection (P<0.05; Fig. 2B). No significant difference in the protein levels of AMFR were observed between the cells in the blank control and scrambled siRNA transfection groups (Fig. 2B).

### siRNA AMFR induces cell cycle arrest at the G0/G1 phase in THP-1 cells

The cell cycle was examined in the THP-1 cells transfected with AMFR-targeting siRNA using flow cytometry with PI staining. AMFR knockdown resulted in disruption of the cell transition between the G0/G1 phase and the S phase and, compared with the untransfected and scrambled siRNA-transfected cells, the percentage of cells in the G0/G1 phase was significantly increased and the percentage of cells in the S phase was significantly decreased in the AMFR siRNA transfected cells (P<0.05). However, there was no significant difference the fraction of cells in the G2/M phase (Fig. 3).

### AMFR siRNA induces THP-1 cell apoptosis

Apoptosis of the THP-1 cells was analyzed using annexin V/PI staining. The results revealed that the percentage of early apoptotic cells increased significantly from 3.88±1.43% of the untransfected THP-1 cells, and 4.01±1.52% of the scrambled siRNA-transfected cells to 19.58±4.29% of the AMFR siRNA-transfected cells (P<0.05; Fig. 4).

### Effects of AMFR knockdown or AFMR-C overexpression on the protein expression levels of ROCK2, cyclin D1 and Bcl-2 in THP-1 cells

AMFR knockdown resulted in significantly decreased protein levels of detectable ROCK2, Bcl-2 and cyclin D1, compared with the untransfected and scrambled siRNA-transfected cells (P<0.05; Fig. 5A), whereas transfection with AMFR-C resulted in significantly increased protein levels of ROCK2, Bcl-2 and cyclin D1, compared with the cells transfected with the pcDNA3.1 plasmid (P<0.05; Fig. 5B).

## Discussion

The expression of AMFR and ROCK2 are reported to correlate with tumor stage and survival rates in types of solid cancer (16–26), and the expression of AMFR is reported to be associated with progression in chronic lymphocytic leukemia (27). In the present study, the effect of AMFR-knockdown and overexpression of AMFR in a cell line, derived from an acute monocytic leukemia patient, which expresses AMFR and ROCK2 (30).

To better understand the function of AMFR, siRNA was used to knockdown the expression of AMFR and a vector was used to induce expression of AMFR-C, a truncated form of AMFR, in the THP-1 human monocytic cell line. Expression of AMFR-C in the THP-1 cells resulted in significantly increased levels of the downstream targets of AMFR (ROCK2, Bcl-2 and cyclin D1). Efficient knockdown of AMFR was also achieved, which inhibited the cell cycle transition between the G0/G1 phase and the S phase, and increased early apoptosis. AMFR knockdown also resulted in decreased levels of detectable ROCK2, Bcl-2 and cyclin D1. The inhibition of the expression of ROCK2 by AMFR has been previously observed in esophageal squamous cell cancer cells (16), indicating that AMFR may affect the expression of ROCK2.

Bcl-2 family proteins are components of the anti-apoptotic machinery and are overexpressed in several types of malignancy, including hematologic malignancies (31). The overexpression of Bcl-2 contributes to cancer progression, inhibits apoptosis and confers resistance to standard anticancer therapies, limiting treatment options for AML (32). RhoC-regulated signals induce apoptosis *in vitro* and *in vivo* via a Bcl-2 dependent pathway (33). In the present study, the overexpression of AMFR-C resulted in increased levels of Bcl-2, whereas downregulation of AMFR led to a significant decrease in the expression of Bcl-2 and increased early apoptosis. These findings suggested that downregulation of Bcl-2 by AMFR suppression may be important role in cell apoptosis.

Cyclin D1 is an initiator and activator of the cell cycle and is overexpressed in a wide range of types of human tumor, includin acute monocytic leukemia (6,7). By co-operating with CDK4/6 kinase, cyclin D1 regulates cell cycle progression, angiogenesis, lipogenesis and mitochondrial function (34). Cyclin D1 is also a key factor in the transition between the G0/G1 and S phases. The present study observed that AMFR-C overexpression resulted in increased levels of cyclin D1, whereas downregulation of AMFR led to a significant decrease in the expression of cyclin D1, and cell cycle progression between the G0/G1 phase and S phase was inhibited. It was concluded that cyclin D1 may be an important component of the AMFR signaling pathway and may be key in cell cycle inhibition.

The results of the present study implicate the AMFR signaling pathway in THP-1 cell proliferation and indicate that ROCK2, Bcl-2 and cyclin D1 may all be involved in this pathway. Whilst the present study involved only one human acute monocytic leukemia cell line, the results suggested that targeting AMFR may present a potential approach for the treatment of acute monocytic leukemia. *In vivo* investigations are Required to confirm these findings and to further elucidate the role of AMFR in acute monocytic leukemia.

## Figures and Tables

**Figure 1:** Protein expression levels of AMFR, AMFR-C and ROCK2 in THP-1 cells or THP-1 cells transfected with pcDNA3.1-AMFR-C. (A) Protein expression levels of AMFR and ROCK2 were detected in the THP-1 cells. (B) AMFR and AMFR-C were detected in the THP-1 cells transfected with 15 *µ*g control plasmid pcDNA3.1 or pcDNA3.1-AMFR-C plasmid, respectively, for 72 h. The protein expression levels were detected using immunoblotting. β-actin was used as the internal reference. AMFR, autocrine motility factor receptor; ROCK, rho-associated, coiled-coil containing protein kinase 2.

**Figure 2:** AMFR siRNA downregulates the mRNA and protein expression levels of AMFR in THP-1 cells. (A) mRNA expression of AMFR at different time-points following transfection with AMFR siRNA, detected using reverse transcription-quantitative polymerase chain reaction. β-actin was used as an internal reference. ^*^P<0.05, vs. blank control; ^#^P<0.05, vs. 72 h. (B) Protein expression of AMFR 72 h after transfection, detected using immunoblotting. β-actin was used as an internal reference. The data are expressed as the mean ± standard deviation of three independent experiments. ^*^P<0.05, vs. blank control; ^#^P<0.05, vs. scrambled siRNA. AMFR, autocrine motility factor receptor; siRNA, small interfering RNA.

**Figure 3:** Effect of AMFR siRNA on THP-1 cell cycle distribution. Cell cycle distribution in THP-1 cells, and THP-1 cells transfected with scrambled siRNA or AMFR siRNA for 72 h were measured using flow cytometry with PI. Data are expressed as the mean ± standard deviation of three independent experiments. ^*^P<0.05, vs. blank control; ^#^P<0.05, vs. scrambled siRNA. AMFR, autocrine motility factor receptor; siRNA, small interfering RNA. PI, propidium iodide.

**Figure 4:** Effect of AMFR siRNA on apoptosis in THP-1 cells. The percentage of early apoptotic cells in the THP-1 cells and the THP-1 cells transfected with scrambled siRNA or AMFR siRNA for 72 h were measured using flow cytometry with annexin V/PI staining. The data are expressed as the mean ± standard deviation of three independent experiments. ^*^P<0.05, vs. blank control; ^#^P<0.05, vs. scrambled siRNA. AMFR, autocrine motility factor receptor; siRNA, small interfering RNA. PI, propidium iodide; FITC, fluorescein isothiocyanate.

**Figure 5:** Effects of AMFR siRNA or pcDNA3.1-AMFR-C on the protein expression levels of ROCK2, Bcl-2 and cyclin D1 in THP-1 cells. (A) Protein expression levels of ROCK2, Bcl-2 and cyclin D1 following AMFR siRNA transfection for 72 h, detected using immunoblotting. ^*^P<0.05, vs. blank control; ^#^P<0.05, vs. scrambled siRNA. (B) Protein expression levels of ROCK2, Bcl-2 and cyclin D1 following transfection with pcDNA3.1-AMFR-C for 72 h, detected using immunobloting. ^*^P<0.05, vs. pcDNA3.1 group. The data are expressed as the mean ± standard deviation of three independent experiments. AMFR, autocrine motility factor receptor; ROCK, rho-associated, coiled-coil containing protein kinase 2; Bcl, B-cell lymphoma.
